The article "The Predictive Value of Neutrophil-Lymphocyte Ratio in Patients with Polycythemia Vera at the Time of Initial Diagnosis for Thrombotic Events" was retracted in 2023. Reasons: unreliable results or conclusions; lack of ethics approval or compliance; concerns about the data; concerns about the peer review.

# The Predictive Value of Neutrophil-Lymphocyte Ratio in Patients with Polycythemia Vera at the Time of Initial Diagnosis for Thrombotic Events

**DOI:** 10.1155/2022/9343951

**Published:** 2022-08-08

**Authors:** Xuekun Wang, Yansong Tu, Mei Cao, Xiaoyan Jiang, Yazhi Yang, Xiaoyan Zhang, Hurong Lai, Huaijun Tu, Jian Li

**Affiliations:** ^1^The Key Laboratory of Hematology of Jiangxi Province, The Department of Hematology, The Second Affiliated Hospital of Nanchang University, 1 Minde Road, Nanchang, 330006 Jiangxi, China; ^2^Graduate School of Medicine, Nanchang University, 465 Bayi Road, Nanchang, 330006 Jiangxi, China; ^3^Faculty of Environment, University of Waterloo, 200 University Avenue, Waterloo, Ontario, Canada N2L 3G1; ^4^Laboratory of Infection & Immunology, School of Basic Medical Sciences, Nanchang University, 465 Bayi Road, Nanchang 330006, China; ^5^The Department of Neurology, The Second Affiliated Hospital of Nanchang University, 1 Minde Road, Nanchang, 330006 Jiangxi, China

## Abstract

**Objective:**

To investigate and discuss the predictive value of the neutrophil-to-lymphocyte ratio (NLR) in patients with polycythemia vera (PV) at the time of initial diagnosis, as well as its clinical significance in predicting the occurrence of thrombotic events and the progression of future thrombotic events during follow-ups, with the goal of providing a reference for the early identification of high-risk PV patients and the early intervention necessary to improve the prognosis of PV patients.

**Method:**

A total of 170 patients diagnosed with PV for the first time were enrolled in this study. The risk factors affecting the occurrence and development of thrombotic events in these patients were statistically analyzed.

**Results:**

NLR (*P* = 0.030), WBC count (*P* = 0.045), and history of previous thrombosis (*P* < 0.001) were independent risk factors for thrombotic events at the time of initial diagnosis. Age ≥ 60 years (*P* = 0.004), NLR (*P* = 0.025), history of previous thrombosis (*P* < 0.001), and fibrinogen (*P* = 0.042) were independent risk factors for the progression of future thrombotic events during follow-ups. The receiver operating characteristic curve (ROC curves) showed that NLR was more effective in predicting the progression of future thrombotic events than age ≥ 60 years, history of previous thrombosis, and fibrinogen. Kaplan-Meier survival analysis showed progression-free survival time of thrombotic events in the high NLR value group (NLR ≥ 4.713) (median survival time 22.033 months, 95% CI: 4.226-35.840), which was significantly lower compared to the low NLR value group (NLR < 4.713) (median overall survival time 66.000 months, 95% CI: 50.670-81.330); the observed difference was statistically significant (*P* < 0.001). The 60-month progression-free survival in the low NLR value group was 58.8%, while it was 32.8% in the high NLR value group.

The article "The Predictive Value of Neutrophil-Lymphocyte Ratio in Patients with Polycythemia Vera at the Time of Initial Diagnosis for Thrombotic Events" was retracted in 2023. Reasons: unreliable results or conclusions; lack of ethics approval or compliance; concerns about the data; concerns about the peer review.

**Conclusion:**

Peripheral blood NLR levels in patients with PV resulted as an independent risk factor for the occurrence of thrombotic events at the time of initial diagnosis and for the progression of future thrombotic events during follow-ups. Peripheral blood NLR levels at the time of initial diagnosis and treatment had better diagnostic and predictive value for the progression of future thrombotic events in patients with PV than age ≥ 60 years, history of previous thrombosis, and fibrinogen.

## 1. Introduction

Polycythemia vera (PV) is a form of myeloproliferative neoplasm (MPN) originating from hematopoietic stem cells. Thrombotic events are a major complication in patients with PV, as well as the most common cause of death [1, 2]. Therefore, early assessment of the risk of occurrence and progression of thrombotic events and early intervention may be effective in improving the prognosis of patients with PV.

By damaging vascular endothelial cells, promoting platelet adhesion and aggregation, and triggering coagulation reactions, inflammation can induce thrombosis, which is more likely to occur with intense inflammation and poor prognosis. White blood cell (WBC) count is an indicator of the systemic inflammatory response that has an important role in thrombosis [3]. One of the risk factors for MPN thrombotic events is the increase and activation of WBC [4].

NLR is the ratio of neutrophils to lymphocytes [5, 6] that has a more significant role in the diagnosis of inflammation and prognosis than the leukocyte subtype alone [7]. In addition to its predictive efficacy in the prognosis of ischemic diseases [8], it has been shown to be strongly associated with thrombotic events in cardiovascular disease [9–11]. Furthermore, a previous study found that the NLR value at the time of initial diagnosis and treatment is a simple-to-calculate marker for systemic inflammation that has better diagnostic and predictive efficacy for future thrombotic event progression in essential thrombocytosis (ET) than other clinical indices [12]. However, there are no relevant studies on the relationship between NLR in PV and thrombotic events in China and abroad. The study of the relationship between NLR and thrombotic events in patients with PV can provide new experimental basis for clinical workers to evaluate the disease and early intervention in the future. In this study, we retrospectively analyzed clinical and laboratory-related parameters in 170 patients with PV, investigated the risk factors for the occurrence and progression of thrombotic events, and analyzed and discussed the correlation between NLR levels and the occurrence and progression of thrombotic events in patients with PV at the time of initial diagnosis and treatment, as well as their clinical significance.

The article "The Predictive Value of Neutrophil-Lymphocyte Ratio in Patients with Polycythemia Vera at the Time of Initial Diagnosis for Thrombotic Events" was retracted in 2023. Reasons: unreliable results or conclusions; lack of ethics approval or compliance; concerns about the data; concerns about the peer review.

## 2. Materials and Methods

### 2.1. Case Information

A total of 170 patients admitted diagnosed with PV for the first time at our hospital between July 2013 and July 2019 were enrolled in this study. Inclusion criteria were as follows: (1) a clear diagnosis of PV, meeting the diagnostic criteria established by WHO in 2008 [13]; (2) patients who were undiagnosed before hospital admission and were not treated with antiplatelet, anticoagulant, or blood cell-lowering related medications. Exclusion criteria were as follows: (1) PV was diagnosed before the patient's admission or patients were treated with antiplatelet, anticoagulant, or hematocrit-lowering related therapy; (2) secondary erythrocytosis; (3) the disease had transformed during follow-ups and the diagnosis met other MPN diagnostic criteria such as ET; (4) the disease had progressed to other types of disease such as primary myelofibrosis, myelodysplastic syndrome, or acute leukemia; (5) the patient had coinfection, tuberculosis, surgery, trauma, malignancy, or the use of immunomodulators or other medications that may affect the blood test.

This study was approved by the Medical Ethics Committee of the Second University Hospital of Nanchang University. Hematocrit is the ratio of red blood cells to the fluid component of your blood or plasma.

Platelets are blood clotting cells that aid in the coagulation of blood. A complete blood count that shows abnormal increases or declines in cell counts may suggest that you have an underlying medical problem that needs to be evaluated further.

### 2.2. Relevant Definitions

Cardiovascular risk factors (CVF) [14]: smoking, hyperlipidemia, diabetes, hypertension, and congestive heart failure. Thrombotic events [15]: arterial thromboembolism refers to acute myocardial infarction, acute ischemic stroke, peripheral arterial disease, and similar. Venous thromboembolism refers to pulmonary embolism, peripheral or visceral venous thrombosis, and similar. Progression of future thrombotic events: a new thrombotic event during follow-up of a patient with no previous history of thrombosis or exacerbation of thrombotic progression at the same site on top of a previous thrombotic event or a new thrombotic event at a different site.

### 2.3. Data Collection

Patient's data in the study were reviewed and collected through the electronic medical record system. All patients were followed up by telephone, outpatient, or inpatient modalities with the future thrombotic event progression as the endpoint of the follow-ups. The last follow-up visit was on September 10, 2019, which included demographic data such as sex, age, cardiovascular risk factors, history of previous thrombosis, future thrombotic event progression, and clinical laboratory findings, such as blood count, biochemistry, coagulation function, JAK2V617F mutation, and bone marrow examination.

The article "The Predictive Value of Neutrophil-Lymphocyte Ratio in Patients with Polycythemia Vera at the Time of Initial Diagnosis for Thrombotic Events" was retracted in 2023. Reasons: unreliable results or conclusions; lack of ethics approval or compliance; concerns about the data; concerns about the peer review.

### 2.4. Breakdown by Group

Patients with PV were divided into a group with and without thrombotic events based on the presence or absence of thrombotic events at the time of the initial consultation. They were separated into two groups: one group had progression of future thrombotic events throughout the follow-up, while the other group did not have progression of future thrombotic events. These groups were determined based on the progression of future thrombotic events. In order to determine the optimal NLR cutoff value, patients were separated into two groups: those with low NLR values and those with high NLR values. These groups were determined using the receiver operating characteristic curve (ROC curve).

### 2.5. Statistical Methods

Data were statistically processed using SPSS 24.0. One-sample Kolmogorov-Smirnov test was used to assess the distribution of the data, and *t*-tests were used for normally distributed measurements. The multifactor analysis was performed using logistic regression for binary outcomes. ROC curves were applied to analyze the predictive value of peripheral blood NLR levels at the time of initial diagnosis and treatment for the occurrence of thrombotic events in patients with PV and to determine the optimal cutoff values with high sensitivity and specificity. Kaplan-Meier analysis was used to assess progression-free survival time to thrombotic events. *P* value of <0.05 was considered to be statistically significant.

## 3. Results

### 3.1. Clinical and Laboratory Test Characteristics

The median age of onset among 170 patients with PV was 56 years (20-83), while 58 patients (34.1%) were aged ≥60 years and 112 (65.9%) <60 years. There were 134 male (78.8%) and 36 female (21.2%) patients, a total of 133 CVF (78.2%) and 37 without CVF (21.8%). In addition, 54 (31.8%) patients had a history of previous thrombosis, and 116 (68.2%) had no previous history of thrombosis; 49 (28.8%) had comorbid diseases with thrombotic events at the time of visit and 121 had no comorbid disease (71.2%) at the time of visit. All 170 patients were tested for the JAK2V617F mutation, among which 107 were positive (62.9%) and 63 were negative (37.1%). The first routine blood test at the time of admission in 170 patients with PV showed a white blood cell count (WBC) of 9.35 ± 5.07 × 10^9^/L, red blood cell count (RBC) 6.61 ± 1.03 × 10^12^/L, hemoglobin count (Hb) 195.28 ± 15.97 g/L, and platelet count (PLT) 281.31 ± 190.13 × 10^9^/L (Table 1).

The article "The Predictive Value of Neutrophil-Lymphocyte Ratio in Patients with Polycythemia Vera at the Time of Initial Diagnosis for Thrombotic Events" was retracted in 2023. Reasons: unreliable results or conclusions; lack of ethics approval or compliance; concerns about the data; concerns about the peer review.

### 3.2. Thrombosis at Initial Diagnosis

At the time of consultation, 49 (28.8%) patients with PV had comorbid diseases with the thrombotic event. The results of the single-factor analysis showed that comorbid disease in thrombosis at the time of initial consultation was closely correlated with NLR (*P* < 0.001), history of previous thrombosis (*P* < 0.001), CVF (*P* = 0.020), and WBC (*P* = 0.006) (Table 2). The multifactorial analysis showed that NLR (*P* = 0.030), WBC (*P* = 0.045), and history of previous thrombosis (*P* < 0.001) were an independent risk factor for the occurrence of thrombotic events at the time of initial diagnosis (Table 3).

### 3.3. Progress of Future Thrombotic Events during Follow-Up

All follow-ups for 170 patients were completed within a median follow-up time of 20.33 (1 to 69) months, and 51 (30.0%) patients progressed to thrombotic events. The single-factor analysis showed that future thrombotic event progression during follow-ups was closely associated with age ≥ 60 years (*P* < 0.001), NLR (*P* < 0.001), WBC (*P* < 0.001), JAK2V617F mutation (*P* = 0.006), history of previous thrombosis (*P* < 0.001), and fibrinogen (FIB) (*P* = 0.011) (Table 4). The multifactorial analysis showed that age ≥ 60 years (*P* = 0.004), NLR (*P* = 0.025), previous thrombosis history (*P* < 0.001), and fibrinogen (*P* = 0.042) were independent risk factors in the progression of future thrombotic events during follow-ups (Table 5). ROC curve analysis showed that the diagnostic efficacy of NLR for the progression of future thrombotic events was more effective than age, history of previous thrombosis, JAK2V61F mutation, and fibrinogen level (AUC NLR > AUC history of previous thrombosis > AUC WBC > AUC age ≥ 60 years AUC JAK2V61F gene mutation > AUC fibrinogen) (Table 6). The sensitivity of the NLR for predicting the progression of thrombotic events was 74.5%, with a specificity of 79.8% when NLR equaled 4.713 (Figure 1).

The 170 followed-up patients were divided into a high NLR group (NLR ≥ 4.713) and a low NLR group (NLR < 4.713). Kaplan-Meier survival analysis showed that the progression-free survival time to thrombotic events in the high NLR group (median overall survival time 22.033 months, 95% CI: 4.226 to 35.840) was significantly lower compared to that in the low NLR group (median overall survival time 66.000 months, 95% CI: 50.670-81.330), and the difference was statistically significant (*P* < 0.001) (see Figure 2). Sixty-month progression-free survival after thrombotic events was 58.8% in the low NLR group. However, the 60-month progression-free survival after thrombotic events in the high NLR group was 32.8%.

The article "The Predictive Value of Neutrophil-Lymphocyte Ratio in Patients with Polycythemia Vera at the Time of Initial Diagnosis for Thrombotic Events" was retracted in 2023. Reasons: unreliable results or conclusions; lack of ethics approval or compliance; concerns about the data; concerns about the peer review.

## 4. Discussion

Recent studies have identified NLR as an essential indicator of immune inflammation [16] that has a wide range of applications. Furthermore, NLR is crucial for the diagnosis and prognosis of infectious diseases. Also, thrombotic events are closely related to noninfectious diseases, such as cardiovascular disease and tumors. However, there are only a few studies on the relationship between NLR and thrombotic events in MPN.

Zhou et al. [12] indicated that a high NLR at the initial diagnosis and treatment is an independent risk factor for future thrombotic events in patients with ET, which suggests that NLR may be related to MPN thrombotic events. Nonetheless, there is no current study on the relationship between NLR and PV thrombotic events. The results of this study indicated that peripheral blood NLR levels at the time of initial diagnosis were not only associated with thrombotic events in patients with PV at the time of initial diagnosis (*P* = 0.030). The high level of NLR at the time of initial diagnosis and treatment indicated a higher risk of combined thrombotic events. Moreover, it had predictive value for the progression of future thrombotic events (*P* = 0.025). In addition, the predictive efficacy in NLR was more significant compared to other indicators. For example, high NLR value indicated shorter survival time in progression-free thrombosis with a higher risk for further development of the original thrombus or new thrombotic events, as well as poor prognosis.

The mechanisms behind NLR and PV thrombotic events are unknown. The process might be analogous to thrombotic events in cardiovascular and tumor disorders [17–22], with NLR acting as an inflammatory-immune signal. There is an increase in neutrophil stress after thrombotic events, indicating an inflammatory response, whereas injured arteries stimulate platelet adhesion and aggregation, triggering a coagulation reaction. On the other hand, lymphocyte stress, which indicates immunological activity, is lowered, lowering immunoprotection and increasing the risk of thrombosis. However, further study is required to fully understand the mechanism.

Age ≥ 60 years has been identified as an independent risk factor for thrombotic events in the conventional thrombotic risk stratification [19]. Patients in this study were divided into two groups based on their age, including ≥60 years and <60 years. The results indicated that even though there was no significant association between age ≥ 60 and PV at the time of initial diagnosis (*P* > 0.05), it was the independent risk factor for future thrombotic event progression in patients with PV (*P* = 0.004). Therefore, it has an important predictive value in patients with PV for future thrombotic event progression, which is consistent with the conventional risk assessment of thrombotic events. Yet, the International Working Group on Myeloproliferative Neoplasms Research and Treatment (IWG-MRT) developed by Tefferi [11] is one of the overall prognostic stratification schemes used in clinical practice for PV based on age (5 points for ≥67 years and 2 points for 57-66 years) that clearly shows the importance of age on the overall prognosis of PV, as well as subdivides the age groups in more detail. The principle is the same, i.e., advanced age is important for the prediction of thrombotic events and overall prognosis in patients with PV.

The article "The Predictive Value of Neutrophil-Lymphocyte Ratio in Patients with Polycythemia Vera at the Time of Initial Diagnosis for Thrombotic Events" was retracted in 2023. Reasons: unreliable results or conclusions; lack of ethics approval or compliance; concerns about the data; concerns about the peer review.

History of thrombosis is not only an independent risk factor in the conventional thrombotic risk stratification in PV patients [23] but a history of venous thrombosis also accumulates points in the IWG-MRT developed by Tefferi [13] in patients with PV. This emphasizes the importance of the history of thrombosis in predicting PV thrombotic events. The results of this study also indicated that a history of thrombosis was not only an independent risk factor for thrombotic events at the time of initial diagnosis (*P* < 0.001) but also an independent risk factor for the progression of future thrombotic events (*P* < 0.001). Although it has been shown that CVF also increases the risk of MPN thrombotic events [24], CVF is not considered as an independent risk factor in the conventional thrombosis risk stratification [23] nor the PV IWG-MRT [15]. Our results revealed no significant correlation between CVF and PV thrombotic events (*P* > 0.05).

The majority of patients with PV have the JAK2V617F mutation [25, 26]. Still, neither the conventional PV thrombosis risk stratification [23] nor the IWG-MRT [13] for PV patients currently includes the JAK2V617F mutation as an independent risk factor. Our results did not reveal the JAK2V617F mutation as an independent risk factor for progression of thrombotic events (*P* > 0.05) in PV patients at the time of initial diagnosis and during the follow-ups; however, there was a significant correlation between JAK2V617F mutations and the thrombotic events during follow-ups (*P* = 0.006) from the single-factor analysis. De Grandis et al. [25] and Lu et al. [27] also found that the JAK2V617F mutation is strongly associated with PV thrombotic events, which suggests that the JAK2V617F mutation might be important for the occurrence of PV thrombotic events at the time of initial diagnosis and in the progression of future thrombotic events.

The article "The Predictive Value of Neutrophil-Lymphocyte Ratio in Patients with Polycythemia Vera at the Time of Initial Diagnosis for Thrombotic Events" was retracted in 2023. Reasons: unreliable results or conclusions; lack of ethics approval or compliance; concerns about the data; concerns about the peer review.

Conventional risk factors for PV thrombosis did not include blood count as an independent risk factor [23], but WBC count > 15 × 10^9^/L accumulates 1 point in the IWG-MRT in PV patients [13]. Our results revealed that WBC was an independent risk factor for the development of PV thrombotic events at the time of initial diagnosis (*P* = 0.045). Even though it was not an independent risk factor for future thrombotic event progression (*P* > 0.05), there was a significant correlation between WBC and future thrombosis progression when analyzed with single-factor analysis (*P* < 0.001). We also found a small number of cases with WBC count > 15 × 10^9^/L (19 cases), while 51 patients had elevated WBC above 10 × 10^9^/L. Therefore, it is hypothesized that the risk of future thrombotic events is increased in PV patients with elevated WBC at the time of initial treatment. Moreover, our results also indicated that RBC and platelet counts were not significantly correlated with the initial thrombotic event or the progression of future thrombotic events (*P* > 0.05).

While neither the conventional risk factors for thrombosis in PV [23] nor the IWG-MRT [13] has included coagulation dysfunction as an independent risk factor for PV, Barraco et al. [28] and Krol [29] have indicated that coagulation dysfunction is an important factor in the development of thrombotic events in PV. Our results did not show a significant correlation (*P* > 0.05) between coagulation function and thrombotic events at the time of initial diagnosis. Still, fibrinogen in coagulation function resulted as an independent risk factor for the progression of thrombotic events during the follow-ups of PV patients (*P* = 0.011).

In the present study, we retrospectively examined the relationship between peripheral blood NLR levels and thrombotic events in patients with PV at the time of initial diagnosis and treatment, finding that NLR is not only an independent risk factor for thrombotic events at initial diagnosis (*P* = 0.030) but also for future thrombotic event progression during follow-ups (*P* = 0.025). The ROC curve also showed that NLR is a stronger predictor of future thrombotic episodes than other factors such as age, past thrombosis history, WBC, and JAK2V617F mutation.

## 5. Conclusion

Peripheral blood NLR levels in patients with PV resulted as an independent risk factor for the occurrence of thrombotic events at the time of initial diagnosis and for the progression of future thrombotic events during follow-ups. Peripheral blood NLR levels at the time of initial diagnosis and treatment had better diagnostic and predictive value for the progression of future thrombotic events in patients with PV than age ≥ 60 years, history of previous thrombosis, and fibrinogen.

The article "The Predictive Value of Neutrophil-Lymphocyte Ratio in Patients with Polycythemia Vera at the Time of Initial Diagnosis for Thrombotic Events" was retracted in 2023. Reasons: unreliable results or conclusions; lack of ethics approval or compliance; concerns about the data; concerns about the peer review.

Therefore, in addition to focusing on factors such as age, previous thrombosis history, blood count, and JAK2V61F mutation in PV patients when assessing the risk of thrombotic events in PV patients, NLR level at the time of initial diagnosis ansd treatment has more clinical significance in predicting the risk of thrombotic events in PV patients. Moreover, these factors may be useful for early assessment and prediction of thrombotic events in patients with PV, early selection of appropriate therapeutic options and prevention, and improved prognosis of patients with PV. The study's border is that it only looked at NLR levels at the time of the first diagnosis and therapy; nevertheless, NLR levels alter over time as illness progresses. Furthermore, because the inflammatory process is complicated, NLR alone is insufficient to determine the amount of inflammatory response. As a result, future research should include baseline levels and dynamics of NLR, as well as other inflammatory markers, to better understand its association to the incidence of PB thrombotic events.

## Figures and Tables

**Figure 1:** ROC curve analysis of age ≥ 60 years, NLR, WBC, JAK2V61F mutation, history of previous thrombosis, and fibrinogen in predicting thrombotic events during follow-up of PV patients.

**Figure 2:** Progression-free survival after thrombotic events' survival rate comparison in the high NLR group and the low NLR group.

**Table 1:** Clinical characteristics of 170 patients with PV at the first consultation.

Categories	Values
Age ≥ 60 years	58
Male	134
History of previous thrombosis	54
JAK2V61F mutation	107
CVF	133
WBC (10^9^/L)	9.35 ± 5.07
RBC (10^12^/L)	6.61 ± 1.03
HB (g/L)	195.28 ± 15.97
PLT (10^9^/L)	281.31 ± 190.13

**Table 2:** Single-factor analysis of risk factors for thrombotic events at initial diagnosis.

Item	Thrombosis group (*n* = 49)	Nonthrombotic group (*n* = 121)	*P* value
Gender, male *n*(%)	37 (75.51)	97 (80.17)	0.501
Age ≥ 60 years *n*(%)	20 (40.82)	38 (31.40)	0.241
JAK2V617F mutation (%)	36 (73.47)	71 (58.68)	0.070
CVF *n*(%)	44 (89.80)	89 (73.55)	0.020
History of thrombosis *n*(%)	41 (83.67)	13 (10.74)	<0.001
NLR	6.602 ± 6.312	4.061 ± 4.131	<0.001
WBC (10^9^/L)	10.527 ± 5.167	8.870 ± 4.977	0.006
RBC (10^12^/L)	6.563 ± 0.965	6.632 ± 1.060	0.832
Hb (g/L)	195.510 ± 16.802	195.190 ± 15.691	0.782
HCT	59.653 ± 5.486	59.148 ± 7.307	0.202
PLT (10^9^/L)	272.220 ± 178.780	285.020 ± 195.179	0.439
Creatinine (*μ*mol/L)	83.535 ± 38.224	77.307 ± 18.908	0.926
Uric acid (*μ*mol/L)	451.397 ± 133.154	439.447 ± 115.753	0.812
eGFR (mL/min)	95.397 ± 38.522	97.528 ± 25.534	0.201
Sodium (mmol/L)	139.016 ± 3.355	138.481 ± 2.703	0.589
Potassium (mmol/L)	4.057 ± 0.608	4.185 ± 0.599	0.220
FIB (g/L)	2.659 ± 0.839	2.573 ± 0.835	0.221
D-dimers (mg/L)	1.558 ± 1.443	1.693 ± 3.248	0.774
APTT (s)	36.045 ± 9.880	36.780 ± 10.143	0.403
PT (s)	13.492 ± 3.585	13.502 ± 3.604	0.561
INR	1.159 ± 0.301	1.151 ± 0.283	0.388
PTA (%)	81.860 ± 26.540	85.493 ± 26.795	0.499
TT (s)	19.420 ± 5.724	19.192 ± 2.161	0.108

The article "The Predictive Value of Neutrophil-Lymphocyte Ratio in Patients with Polycythemia Vera at the Time of Initial Diagnosis for Thrombotic Events" was retracted in 2023. Reasons: unreliable results or conclusions; lack of ethics approval or compliance; concerns about the data; concerns about the peer review.

**Table 3:** Multifactorial analysis of risk factors for thrombotic events at the time of initial diagnosis.

Variant	*P* value	OR	95% CI
NLR	0.030	1.192	1.017-1.398
WBC	0.045	0.869	0.758-0.997
History of thrombosis	<0.001	48.912	16.797-142.429
CVF	0.435	1.701	0.449-6.449

**Table 4:** Single-factor analysis of risk factors for progression to future thrombotic events.

Item	Thrombosis group (*n* = 51)	Nonthrombotic group (*n* = 119)	*P* value
Gender, male *n*(%)	36 (70.59)	98 (82.35)	0.085
Age ≥ 60 years *n*(%)	33 (64.71)	25 (21.01)	<0.001
JAK2V617F mutation *n*(%)	40 (78.43)	67 (56.30)	0.006
CVF *n*(%)	39 (76.47)	94 (78.99)	0.715
History of thrombosis *n*(%)	36 (70.59)	18 (15.13)	<0.001
NLR	8.174 ± 7.346	3.344 ± 2.353	<0.001
WBC (10^9^/L)	12.259 ± 5.926	8.099 ± 4.092	<0.001
RBC (10^12^/L)	6.589 ± 1.071	6.622 ± 1.019	0.904
Hb (g/L)	196.120 ± 18.938	194.920 ± 14.589	0.723
HCT	59.775 ± 6.070	59.087 ± 7.131	0.115
PLT (10^9^/L)	306.250 ± 176.270	270.530 ± 195.553	0.120
Creatinine (*μ*mol/L)	82.041 ± 37.003	77.843 ± 19.592	0.735
Uric acid (*μ*mol/L)	445.692 ± 135.430	441.691 ± 114.472	0.938
eGFR (mL/min)	94.897 ± 37.700	97.778 ± 25.753	0.230
Sodium (mmol/L)	138.502 ± 3.515	138.692 ± 2.617	0.199
Potassium (mmol/L)	4.143 ± 0.609	4.151 ± 0.602	0.909
FIB (g/L)	2.895 ± 1.164	2.471 ± 0.606	0.011
D-dimers (mg/L)	2.479 ± 4.897	1.301 ± 0.999	0.059
APTT (s)	37.666 ± 12.108	36.098 ± 9.035	0.661
PT (s)	13.727 ± 3.847	13.401 ± 3.483	0.833
INR	1.187 ± 0.318	1.151 ± 0.283	0.975
PTA (%)	80.302 ± 27.010	86.222 ± 26.473	0.293
TT (s)	19.917 ± 5.588	18.975 ± 2.144	0.243

**Table 5:** Multifactorial analysis of risk factors for the progression of future thrombotic events.

Variant	*P* value	OR	95% CI
Age ≥ 60 years	0.004	4.378	1.614-11.873
NLR	0.025	1.279	1.032-1.587
History of thrombosis	<0.001	11.604	4.463-30.173
Fibrinogen	0.042	1.820	1.023-3.238
WBC	0.675	0.970	0.841-1.118
JAK2V617F mutation	0.767	1.179	0.396-3.508

**Table 6:** ROC curve analysis of aged ≥60 years, NLR, WBC, JAK2V61F gene mutation, history of previous thrombosis, and fibrinogen in predicting thrombotic events during follow-up of PV patients.

Variant	Area under the curve	*P* value	95% CI
NLR	0.813	<0.001	0.743-0.883
History of thrombosis	0.777	<0.001	0.695-0.860
WBC	0.757	<0.001	0.677-0.837
Age ≥ 60 years	0.718	<0.001	0.630-0.806
JAK2V61F mutation	0.611	0.022	0.521-0.700
Fibrinogen	0.584	0.083	0.482-0.687

The article "The Predictive Value of Neutrophil-Lymphocyte Ratio in Patients with Polycythemia Vera at the Time of Initial Diagnosis for Thrombotic Events" was retracted in 2023. Reasons: unreliable results or conclusions; lack of ethics approval or compliance; concerns about the data; concerns about the peer review.

## Data Availability

The datasets used and analyzed during the current study are available from the corresponding author on reasonable request.

## References

[1] Tefferi A., Barbui T. (2019). Polycythemia vera and essential thrombocythemia: 2019 update on diagnosis, risk-stratification and management. *American Journal of Hematology*.

[2] Matos M. F. (2011). The role of IL-6, IL-8 and MCP-1 and their promoter polymorphisms IL-6 -174GC, IL-8 -251AT and MCP-1 -2518AG in the risk of venous thromboembolism: A case- control study. *Thrombosis Research*.

[3] Reganon E., Vila V., Martínez-Sales V. (2007). Sialic acid is an inflammation marker associated with a history of deep vein thrombosis. *Thrombosis Research*.

[4] Sun T., Zhang L. (2013). Thrombosis in myeloproliferative neoplasms with JAK2V617F mutation. *Clinical & Applied Thrombosis/hemostasis*.

[5] Arbel Y., Finkelstein A., Halkin A. (2012). Neutrophil/lymphocyte ratio is related to the severity of coronary artery disease and clinical outcome in patients undergoing angiography. *Atherosclerosis*.

[6] Alazzam M. B., Al-Radaideh A. T., Binsaif N., AlGhamdi A. S., Rahman M. A. (2022). Advanced deep learning human herpes virus 6 (HHV-6) molecular detection in understanding human infertility. *Computational Intelligence and Neuroscience*.

[7] Sabri G. (2014). Platelet/lymphocyte ratio and risk of in-hospital mortality in patients with ST-elevated myocardial infarction. *Medical Science Monitor: International Medical Journal of Experimental and Clinical Research*.

[8] Celikbilek A., Ismailogullari S., Zararsiz G. (2014). Neutrophil to lymphocyte ratio predicts poor prognosis in ischemic cerebrovascular disease. *Journal of Clinical Laboratory Analysis*.

[9] Xu N., Tang X. F., Yao Y. (2018). Predictive value of neutrophil to lymphocyte ratio in long-term outcomes of left main and/or three-vessel disease in patients with acute myocardial infarction. *Catheterization and Cardiovascular Interventions*.

[10] Alazzam M. B., Mansour H., Alassery F., Almulihi A. (2021). Machine learning implementation of a diabetic patient monitoring system using interactive E-App. *Computational Intelligence and Neuroscience*.

[11] Zhai M., Wang J., Yu L., Fu X., Li L. (2017). Predictive value of neutral granulocyte to lymphocyte ratio on the prognosis of patients with acute cerebral infarction. *Chinese Journal of Cerebrovascular Disease*.

The article "The Predictive Value of Neutrophil-Lymphocyte Ratio in Patients with Polycythemia Vera at the Time of Initial Diagnosis for Thrombotic Events" was retracted in 2023. Reasons: unreliable results or conclusions; lack of ethics approval or compliance; concerns about the data; concerns about the peer review.

[12] Zhou D., Cheng H., Chen W., Li Z., Xu K. (2019). Relationship between peripheral thromboplastin ratio and thrombotic events in primary thrombocytopenic patients at the time of initial diagnosis and treatment. *Chinese Journal of Experimental Hematology*.

[13] Shi Z., Xiao Z. (2016). Interpretation of the Chinese expert consensus on the diagnosis and treatment of true erythrocytosis (2016 edition). *Chinese Journal of Hematology*.

[14] Marchioli R., Finazzi G., Landolfi R. (2005). Vascular and neoplastic risk in a large cohort of patients with polycythemia vera. *Journal of Clinical Oncology*.

[15] Barbui T., Finazzi G., Carobbio A. (2012). Development and validation of an international prognostic score of thrombosis in World Health Organization-essential thrombocythemia (IPSET-thrombosis). *Blood*.

[16] Zhu J., Zhu L., Yin Y., Ruan Z. (2014). Peripheral blood NLR changes in patients with early ventricular arrhythmias in acute myocardial infarction and their significance. *Shandong Medical*.

[17] Alazzam M. B., Tayyib N., Alshawwa S. Z., Ahmed M. K. (2022). Nursing care systematization with case-based reasoning and artificial intelligence. *Journal of Healthcare Engineering*.

[18] Ferroni P., Riondino S., Formica V. (2015). Venous thromboembolism risk prediction in ambulatory cancer patients: clinical significance of neutrophil/lymphocyte ratio and platelet/lymphocyte ratio. *International Journal of Cancer*.

[19] He J., Li J., Wang Y., Hao P., Hua Q. (2014). Neutrophil-to-lymphocyte ratio (NLR) predicts mortality and adverse-outcomes after ST-segment elevation myocardial infarction in Chinese people. *International Journal of Clinical and Experimental Pathology*.

[20] Xu L., Tao B. (2017). Correlation of neutrophil lymphocyte ratio and acute myocardial infarction. *China Cardiovascular Research*.

[21] Carobbio A., Vannucchi A. M., De Stefano V. (2022). Neutrophil-to-lymphocyte ratio is a novel predictor of venous thrombosis in polycythemia vera. *Blood Cancer Journal*.

[22] Huang B. (2012). Regulation of immunity and inflammation in the tumor microenvironment. *Chinese Journal of Cancer Biotherapy*.

[23] Barbui T., Barosi G., Birgegard G. (2011). Philadelphia-negative classical myeloproliferative neoplasms: critical concepts and management recommendations from European LeukemiaNet. *Journal of Clinical Oncology*.

[24] Casini A., Fontana P., Lecompte T. P. (2013). Thrombotic complications of myeloproliferative neoplasms: risk assessment and risk-guided management. *Journal of Thrombosis and Haemostasis*.

[25] De Grandis M., Cambot M., Wautier M. P. (2013). JAK2V617F activates Lu/BCAM-mediated red cell adhesion in polycythemia vera through an EpoR-independent Rap1/Akt pathway. *Blood*.

The article "The Predictive Value of Neutrophil-Lymphocyte Ratio in Patients with Polycythemia Vera at the Time of Initial Diagnosis for Thrombotic Events" was retracted in 2023. Reasons: unreliable results or conclusions; lack of ethics approval or compliance; concerns about the data; concerns about the peer review.

[26] Elbadry M. I., Tawfeek A., Abdellatif M. G. (2022). Unusual pattern of thrombotic events in young adult non-critically ill patients with COVID-19 may result from an undiagnosed inherited and acquired form of thrombophilia. *British Journal of Haematology*.

[27] Lu W. J., Lin K. C., Huang S. Y. (2014). Role of a Janus kinase 2-dependent signaling pathway in platelet activation. *Thrombosis Research*.

[28] Barraco D., Cerquozzi S., Hanson C. A. (2017). Prognostic impact of bone marrow fibrosis in polycythemia vera: validation of the IWG-MRT study and additional observations. *Blood Cancer Journal*.

[29] Kroll M. H., Michaelis L. C., Verstovsek S. (2015). Mechanisms of thrombogenesis in polycythemia vera. *Blood Reviews*.

